The article "Effects of Aerobic Exercise on Sleep Quality and Mental Health of College Students" was retracted in 2023. Reasons: signs of a paper mill; suspected computer-generated content; unreliable results or conclusions; lack of ethics approval or compliance.

# Effects of Aerobic Exercise on Sleep Quality and Mental Health of College Students

**DOI:** 10.1155/2022/8366857

**Published:** 2022-10-10

**Authors:** Lu Li

**Affiliations:** Tangshan Polytechnic College, Tangshan, Hebei 063299, China

## Abstract

**Objective:**

In recent years, people's living standards have been greatly improved, but at the same time, it also brings many health problems, among which mental health problems and sleep problems of college students are important problems. The aim of the study is to explore the effect of physical activity intervention on college students' mental health and provide a new way of thinking for colleges and universities to carry out mental health interventions.

**Methods:**

This paper focuses on the physical health problems of college students and explores the relationship between aerobic exercise, emotion, and sleep quality among college students. The SPSS statistical method was used to analyze the differences in aerobic exercise, emotion, and sleep quality among college students in terms of demographic variables; to explore the relationship between aerobic exercise, emotion, and sleep quality; and to construct a structural equation model using the relationship between them. *Results/Discussion*. This study explores the relationship between aerobic exercise and sleep quality and psychological health of college students, further analyzes the path model of the role of aerobic exercise and psychological health on sleep quality of college students, and verifies it through experiments, which proves to help universities and relevant departments understand the current situation of exercise and sleep quality of college students and provide timely and effective design of mandatory aerobic exercise courses for college students who lack exercise and have sleep problems. At the same time, it helps college students to understand their sleep situation and adjust their aerobic exercise courses according to their sleep status.

## 1. Introduction

Sleep is both a physiological regulatory process of the nervous system and the most basic human need. A high level of sleep quality allows individuals to recover energy and stamina, improve the body's metabolic capacity, promote organism growth, consolidate memory, and enhance individual cognitive function, while insomniacs are often accompanied by a sense of unrecovered waking, fatigue, memory loss, lack of concentration, and abnormal emotions, leading to a decline in their quality of life, work, or study efficiency. At this stage, social college students are facing various aspects of stress and poor inhibitory control, which makes them prone to mental health and sleep quality problems. Inhibitory control ability is the ability to inhibit internal dominant responses or external irrelevant responses to enable oneself to adapt to conflicts, and it includes active inhibitory control and reactive inhibitory control [1]. Good inhibitory control is a guarantee of rational behavior in individuals, and once inhibitory control is impaired, it can induce a variety of problems, such as depression, schizophrenia, and attention deficit hyperactivity disorder. Therefore, improving inhibitory control is extremely important for individual development. It has been shown that exercise can effectively promote the development of inhibitory control. The effect of exercise on inhibitory control may be influenced by the intensity of exercise. It was found that exercise of different intensities improved inhibitory control, but moderate intensity improved better than the high-intensity and low-intensity groups [2]. It has also been found that high-intensity exercise interventions impaired inhibitory control in individuals, as well as no positive effect on inhibitory control, were observed after low-intensity exercise interventions, but the improvement of inhibitory control by moderate-intensity exercise was generally confirmed. In the existing studies on sleep quality, most of them focus on the change of individual mood after sleep quality improvement or the effect of individual mood state on sleep quality, but less on the relationship between aerobic exercise, mood, and sleep quality in college students.

The article "Effects of Aerobic Exercise on Sleep Quality and Mental Health of College Students" was retracted in 2023. Reasons: signs of a paper mill; suspected computer-generated content; unreliable results or conclusions; lack of ethics approval or compliance.

The literature [3] studied mice in a chronic unpredictable mild stress depression model, trained with treadmill running as an antidepressant, and the experimental results showed that the training not only reduced depression but also improved olfactory discrimination and sensitivity (threshold), and further molecular biological results showed that exercise promoted neuronal activity and prevented the neuronal loss in the hippocampus. In conclusion, exercise can reduce depressive symptoms in mice by improving neuronal function and activity. Also in the literature [4], 30 obese adolescents aged 12-17 years were selected as subjects for a study to implement a planned, structured, and time-specific aerobic exercise intervention and to test their academic ability, social ability, motor ability, body image, and self-esteem indicators. Good inhibitory control is a guarantee of rational behavior in individuals, and when inhibitory control is impaired, it can induce a variety of problems, such as depression, schizophrenia, and attention deficit hyperactivity disorder. Therefore, improving inhibitory control is extremely important for individual development. It has been shown that motor exercise can effectively promote the development of inhibitory control. Results revealed significant pre- and postimprovements in body image, academic ability, and social competence, thus suggesting that aerobic exercise can promote improvements in body image, academic performance, and social competence in obese adolescents and is also associated with improvements in psychological status. In the literature [5], a 3-month boxing aerobic exercise training program was designed for adolescents with mental health problems. Instead, it was found that there were no significant changes in human physiological indicators such as weight and BMI, but it had a positive effect on the improvement of their mental health status, allowing the adolescents to increase their self-confidence, improve their physical fitness as well as their academic performance, and start to be willing to contact and participate in campus activities.

The article "Effects of Aerobic Exercise on Sleep Quality and Mental Health of College Students" was retracted in 2023. Reasons: signs of a paper mill; suspected computer-generated content; unreliable results or conclusions; lack of ethics approval or compliance.

There are many ways to improve sleep problems, such as drug therapy, physical therapy (transcranial magnetism, brain wave therapy, etc.), and exercise interventions. Pharmacological interventions are more effective, but they are not easily used because of the side effects of sleeping pills and the tendency to form drug dependence. Physiotherapy is not the best way to improve sleep quality because it is effective and has few side effects, but it requires the guidance of a specialist and some financial support. Aerobic exercise is more suitable for all types of people than the above-mentioned therapies, and it is convenient and quick. In addition to improving sleep quality, aerobic exercise can also strengthen an individual's immune system and improve their mood. Aerobic exercise is a kind of sports designed to improve the basic quality of individuals, strengthen the nervous system, and regulate emotional ability, and it is also a long time, planned, and regular low-intensity exercise, which can have a positive impact on the individual's cognition, emotion, and behavior. Therefore, aerobic exercise is becoming an important tool for individuals to improve their sleep quality. The introduction of mandatory aerobic exercise courses at universities is also inextricably linked to the quality of sleep and mental health of college students.

This study has more important theoretical significance. The current research on sleep quality at home and abroad is mostly focused on the changes in physiological and psychological indicators after the improvement of individual sleep quality, but the research on the antecedent influence mechanism of sleep quality is not systematic and comprehensive enough [6]. In this study, we will investigate the objective and subjective factors affecting individual sleep quality and understand the current situation of aerobic exercise, emotion, and sleep quality among college students and the relationship between the three variables, to provide a theoretical basis for the relevant departments of colleges and universities to strengthen the physical exercise of college students and intervene in their sleep problems. Sleep inventory applies to a wide range of populations and monitors sleep habits, sleep quality, and sleep hygiene issues. The Sleep Disorders Scale, on the other hand, is designed to detect insomnia, respiratory-related sleep disorders, and circadian sleep rhythm disorders and applies to a narrower population. The relationship between aerobic exercise, as a common way for individuals to release stress and relieve mental tension, and sleep quality may be directly or indirectly influenced by mediating or moderating variables. Emotions are an important psychological characteristic of individuals, and individuals are highly likely to awaken emotions and process them during the process of entering aerobic exercise, which further affects the quality of sleep.

The article "Effects of Aerobic Exercise on Sleep Quality and Mental Health of College Students" was retracted in 2023. Reasons: signs of a paper mill; suspected computer-generated content; unreliable results or conclusions; lack of ethics approval or compliance.

Therefore, this study explores the mechanism of the effect of aerobic exercise and emotion on sleep quality from a new perspective, taking into account the characteristics of the times, and elaborates on the relationship between aerobic exercise and sleep quality in college students. This study also has important practical value. As an important part of life, aerobic exercise plays an important role in improving the physical and mental health of individuals. Therefore, this study explores the relationship between aerobic exercise and sleep quality among college students and further analyzes the path model of the role of aerobic exercise and emotion on sleep quality among college students. At the same time, it helps college students understand their sleep situation and make self-adjustment for their sleep conditions.

## 2. Methods

### 2.1. Evaluation Criteria

Most scholars believe that sleep quality mainly consists of two parts: subjective sleep quality and objective sleep quality. Therefore, the existing assessment tools on sleep quality are mainly divided into two categories: subjective sleep quality assessment tools and objective sleep quality assessment tools. In terms of subjective measures, individuals mainly self-rate their sleep quality using self-assessment scales. Sleep scales are commonly used not only in basic research but also in clinical screening for sleep-related problems. Depending on the content and scope of the sleep scale, researchers have subdivided the sleep scale into the Comprehensive Sleep Scale and the Sleep Disorders Scale. The comprehensive sleep inventory applies to a wide range of populations and monitors sleep habits, sleep quality, and sleep hygiene problems. The Sleep Disorders Scale, on the other hand, is designed to detect insomnia, breathing-related sleep disorders, and circadian sleep rhythm disorders and applies to a narrower population [7].

The article "Effects of Aerobic Exercise on Sleep Quality and Mental Health of College Students" was retracted in 2023. Reasons: signs of a paper mill; suspected computer-generated content; unreliable results or conclusions; lack of ethics approval or compliance.

Due to the complexity and multidimensionality of the sleep quality structure, as well as the limitations of research and development costs, the assessment tools on sleep quality are mainly characterized as follows: basic research mainly uses subjective assessment tools, while clinical diagnosis mainly uses objective assessment tools. However, it is believed that the future research trend will be a combination of subjective and objective measurement tools to assess the sleep quality of individuals more accurately and scientifically. The compulsory aerobics courses in colleges and universities can set diversified types of sports according to the demographic characteristics of students so that college students can make diversified choices according to their conditions. In addition, relevant departments of colleges and universities should also actively promote extracurricular sports and carry out regular or irregular sports activities to encourage college students to integrate into the group and relieve the pressure of study and interpersonal aspects. According to the PSQI classification criteria, the total score of 28 is the critical point for assessing individual sleep quality; i.e., the quality of individual sleep can be determined according to the critical value combined with Table 1; it can be seen that the total mean PSQI score of college students in this study is 16.25 ± 3.16, which shows that the overall sleep quality of college students today is poor [8]. In addition, Table 1 also shows that the total PSQI score and the sleep onset time, sleep efficiency, subjective sleep quality, daytime dysfunction, and sleep disorder factor scores are higher than the reference values provided by the revisers of the Chinese version of the PSQI.

Mental health refers to a person's physical and mental health in an excellent state, which includes normal intellectual development, optimistic emotions, the firm will, accurate behavior, sufficient energy, good strain, ability to adapt to the external environment, ability to face daily life with ease and comfort and maintain abundant work energy, courage to undertake, good interpersonal relationship, physical age in line with mental age, and ability to look forward to the future [9]. Internet information updates, the rapid development of new media, the rhythm of knowledge updates, multiple changes in the external environment, family factors, and self-psychological adjustment ability are all factors that affect mental health problems. Mental health refers to a balanced relationship between the subjective world and the objective environment of a person and a good interpersonal relationship between the self and others to maintain, that is, not only to obtain ensure a sense of self-security but also to achieve self-worth, with the ability to provide help for the health of others.

The article "Effects of Aerobic Exercise on Sleep Quality and Mental Health of College Students" was retracted in 2023. Reasons: signs of a paper mill; suspected computer-generated content; unreliable results or conclusions; lack of ethics approval or compliance.

### 2.2. Methods

All students in the experimental group were firstly signed in, and then, they carried out aerobic exercise activities such as ball games, gymnastics, fitness, and endurance exercises, according to their interests. Steps were required to reach more than 6000 steps per activity. In the intervention, emphasis was placed on exercise, humanization, sustainability, and scientific communication to reduce the psychological resistance of the subjects in the intervention process; excluding negative influences and other interference, the control group did not have any intervention, and the students carried out their normal study life according to their habits [10]. The mental health aspects of college students before and after the physical activity intervention were measured using the Symptom Self-Rating Scale SCL-90 mental health test scale, and the test was conducted in two sessions, one before the physical activity intervention and another after the experimental intervention.

### 2.3. Principle

A single exercise round has been shown to induce plasticity-promoting effects at both the molecular and systemic levels and to lead to arousal as well as increased cerebral blood flow. Aerobic exercise also affects neurophysiological pathways, with improved performance on various cognitive task categories, such as attention, working memory, and executive function, while acute aerobic exercise has the most pronounced positive effects on executive function, a higher cognitive function that controls individual thoughts and actions, and thus, acute aerobic exercise is considered an effective strategy for executive function. The structure and function of the prefrontal cortex (PFC) are related to executive function, and therefore, changes in activation of PFC regions are associated with exercise-induced improvements in cognitive performance. The left and right dorsolateral prefrontal cortex (DLPFC) is highly active in response to recall and mental effort. The left DLPFC is associated with processing speed and executive function and appears to be influenced by acute exercise. Enhanced cognitive function after exercise is associated with greater activation of the DLPFC, which suggests increased attention or mental focus after exercise [11]. For example, in a postexercise cognitive test in healthy adults, a single 30-second session of high-intensity cycling until exhaustion increased DLPFC activity. Similarly, 10 minutes of moderate-intensity exercise at 50% maximal oxygen consumption (VO2Max) was effective in activating the left DLPFC. Studies have also been conducted on brain area activation in the flanker task during acute aerobic loading, with the site of activation in the L-DLPFC, and there has been considerable research on the potential mechanisms of PFC activation leading to improved brain function within minutes of exercise. Considerable research has been conducted on the potential mechanisms of PFC activation leading to improved brain function within minutes after exercise. During low to moderate intensity exercise, cerebral blood flow and oxygenation levels are increased, which may promote nutrient distribution throughout the brain and induce arousal during subsequent cognitive tests. As shown in Figure 1, the association between aerobic exercise and physical and mental health is mapped.

The article "Effects of Aerobic Exercise on Sleep Quality and Mental Health of College Students" was retracted in 2023. Reasons: signs of a paper mill; suspected computer-generated content; unreliable results or conclusions; lack of ethics approval or compliance.

As exercise reaches higher intensities, resources are shifted from cognitive processing areas (including the PFC) to motor function areas of the brain. This response is known as transient subfrontal voxels and may lead to downstream cognitive improvements in later mental tasks due to reperfusion of cortical areas. At low levels of exercise, brain activity is limited and does not receive proper neuronal activation, and arousal levels are low; whereas at moderate levels of aerobic exercise, arousal levels increase and become optimal; when arousal is further increased, neurons that are not part of this pattern are also activated, producing neural “noise” that leads to cognitive performance decreases [12]. Basic research has mainly used subjective assessment tools, while the clinical diagnosis has mainly used objective assessment tools. However, it is believed that the future research trend will be a combination of subjective and objective measurement tools to assess the sleep quality of individuals more accurately and scientifically. It has been supported by meta-analyses that moderate aerobic exercise improves cognitive performance more than light or high-intensity exercise: the level of arousal from moderate exercise is an important condition for improved cognitive performance. However, activation of motor areas at higher intensities impairs activation of the prefrontal cortex, which negatively affects cognitive performance. Another hypothesis suggests that neurotransmitters produced by moderate-intensity exercise promote cognitive performance, whereas catecholamines produced by high-intensity exercise hurt cognition. The pattern of cortical activation of motor responses also depends on movement pattern, rhythm, and type of muscle contraction. Movement pattern and intensity preference reflect changes in cortical electrical activation following exercise; high-intensity exercise (80% maximal power output) leads to reduced frontal beta activity in the preferred exercise (running) but not in other movement patterns (cycling and rocking arm) [13]. All these results will support that changes in prefrontal cortical brain responses reflect functional (cognitive and emotional) processes during exercise, dependent on dose-response relationships, and individual exercise preferences.

The article "Effects of Aerobic Exercise on Sleep Quality and Mental Health of College Students" was retracted in 2023. Reasons: signs of a paper mill; suspected computer-generated content; unreliable results or conclusions; lack of ethics approval or compliance.

In conclusion, studies comparing the effects of specific exercise intensities on executive function have yielded inconsistent results. When investigating the effects of more than one exercise intensity, most studies support greater improvements in executive function following moderate aerobic exercise. Furthermore, the previous comprehensive literature supports that exercise intensity is the primary moderator of the effects of acute aerobic exercise on executive control, with moderate-intensity aerobic exercise being the most beneficial for higher cognitive function.

### 2.4. Research Subjects

In this study, 760 college students were surveyed by multistage quota sampling method, 760 questionnaires were distributed, 734 questionnaires were collected, and 719 valid questionnaires were obtained after eliminating regular responses and incomplete questionnaires (questionnaires with missing values of 15 questions or more were considered incomplete), with an effective rate of 98.1%. The specific distribution of subjects is shown in Table 2.

After the questionnaires were uniformly collected, the data were entered using SPSS 7.0 and analyzed as follows: descriptive statistics, independent samples *t*-test, one-way ANOVA, correlation analysis, and regression analysis, as well as mediating effects, test using SPSS 7.0, and then model path analysis of the data using Amos 21.0.

### 2.5. Statistical Analysis

After applying FC-NIRS to complete the calculation of FC measured before and after the exercise intervention, the experimental data were statistically analyzed through the MATLAB data platform [14]. Among them, the comparative analysis was performed by applying independent samples *t*-test or nonparametric test for comparative information between groups; one-way ANOVA was used for intensity factors to determine whether the acute aerobic exercise of different exercise intensities had different effects on resting-state functional connectivity of college students; the cortical R SFC total means were analyzed using an analysis of covariance to determine whether acute aerobic exercise had different effects on RSFC in college students at different exercise levels; next, a paired samples *t*-test was used between the pretest and posttest data for each group to determine whether there was a significant change in RSFC; next, for each subject and each test, Pearson correlation coefficients were calculated for the time course of each two channels to produce a correlation matrix. The significance level was set at *P* < 0.05.

The article "Effects of Aerobic Exercise on Sleep Quality and Mental Health of College Students" was retracted in 2023. Reasons: signs of a paper mill; suspected computer-generated content; unreliable results or conclusions; lack of ethics approval or compliance.

## 3. Results

### 3.1. Mental Health

Using the SPSS software package, 760 college students who participated in the questionnaire survey were analyzed by statistical and correlation processing. The results are shown in Table 3. Among the male college students, the scores of compulsive symptoms, interpersonal sensitivity, depression, hostility, and paranoia reflecting mental health levels were higher than the scores of SCL-90 factors of the national college students [15]. In the gender differences between males and females, the total SCL-90 scores and factor scores of female college students were higher than those of male college students, and the mental health problems of female college students were more serious than those of male college students.

Both male and female subjects had high data of every single index of mental health level, and the scores of test factors exceeded the SCL-90 scores of college students' norm, and the total scores of SCL-90 were > 160. The factors of obsessive-compulsive symptoms, interpersonal sensitivity, and depression are the main mental health problems of female students. In comparison with male students than female students, male students have lower mean scores in SCL-90 total and factor scores than female students, and from the overall perspective, both male and female students have higher SCL-90 total scores as well as factor scores than college students' normative SCL-90 factor scores [16].

Through the opportunity of aerobic exercise, many students will take the initiative to talk and communicate with the opposite sex; make friends with others with sincerity, so the score of interpersonal sensitivity and paranoia is reduced; release their depressed mood through physical activity; and reduce the score of depression factor. Through aerobic exercise, college students' psychological confidence is increased; attention is shifted, and the score of anxiety factor is reduced, from the overall. In the overall analysis, the mental health level of female students and the total SCL-90 scores were higher than those of male students, which proved that the mental health level of female students was lower than that of male students after the experimental intervention [17].

The article "Effects of Aerobic Exercise on Sleep Quality and Mental Health of College Students" was retracted in 2023. Reasons: signs of a paper mill; suspected computer-generated content; unreliable results or conclusions; lack of ethics approval or compliance.

### 3.2. Inhibitory Control Capability

As shown in Figure 2, the growth rates of response time in the inconsistent and consistent conditions were 3.65% and 3.95% for the daily exercise group and 2.82% and 2.34% for the every-other-day exercise group in the inconsistent and consistent conditions, respectively, indicating that the response inhibition ability of college students in the middle and late stages of the aerobic exercise intervention was in a slow growth phase. The growth rates of response time in the inconsistent and consistent conditions were 1.75% and 4.53% for the daily exercise group and 3.59% and 0.83% for the every-other-day exercise group in the inconsistent and consistent conditions, respectively, indicating a slow growth phase of response inhibition for college students in the middle and late stages of the aerobic exercise intervention.

No significant changes in the accuracy of either response inhibition ability or active inhibition ability (consistent and inconsistent conditions) were found in the middle to late stages of the 4-week moderate-intensity aerobic exercise intervention, and no differences were found in response time. Aerobic exercise is a kind of sport designed to improve the basic quality of individuals, strengthen the nervous system, and regulate emotional ability, and it is also a long, planned, and regular low-intensity exercise that can have a positive impact on individuals' cognition, mood, and behavior. This suggests that there were no large changes in inhibitory control ability in college students during the middle to late stages of the 4-week moderate-intensity aerobic exercise intervention. In addition, our study went on to compare the effects of two different exercise frequencies, daily and every other day, on inhibitory control in college students, but the results still did not reveal differences, suggesting that daily and every-other-day exercises were equally effective in promoting the development of inhibitory control in the middle and late stages of the aerobic exercise intervention [18]. The subjects' response inhibition ability (consistent and inconsistent conditions) showed little change in correctness, while response time showed a rapid decrease with an increasing number of interventions. This suggests that response inhibition is in a rapid improvement phase early in the aerobic exercise intervention. Individuals learning new motor skills require the involvement of the cerebellum, which can also facilitate connections between the brain and cerebellum, thereby enhancing the development of brain function [19]. Previous studies have shown that the cerebellum also has a crucial role in the cognitive functions of individuals, such as inhibition and memory functions. Similarly, the cerebellum is heavily involved when learning new skills, and there is a period of rapid improvement after repeated connections in the prelearning period, and inhibitory control is also a part of brain function that improves rapidly after long-term aerobic exercise interventions.

The article "Effects of Aerobic Exercise on Sleep Quality and Mental Health of College Students" was retracted in 2023. Reasons: signs of a paper mill; suspected computer-generated content; unreliable results or conclusions; lack of ethics approval or compliance.

### 3.3. Sleep Quality

As shown in Table 4, the amount of aerobic exercise among college students was negatively correlated with the total PSQI score and five factors: time to sleep, daytime dysfunction, sleep disturbance, subjective sleep quality, and sleep efficiency. The amount of aerobic exercise in college students' mental health was positively correlated. In addition, from Table 4, it was also found that college student's mental health was negatively correlated with total PSQI score and four factors of time to sleep, subjective sleep quality, sleep efficiency, and daytime dysfunction; college students' negative mood was positively correlated with total PSQI score and factors of time to sleep, daytime dysfunction, sleep duration, sleep disorder, subjective sleep quality, and hypnotic drugs [20].

Regression analyses were performed on the quantities to explore the mechanisms influencing sleep quality among college students. Since the demographic variables were all categorical variables, they were virtualized into continuous variables before control [21]. Also, to avoid the problem of multicollinearity, aerobic exercise, mood, sleep quality, and the control variables were standardized in this study and later analyzed according to the stepwise test procedure for mediating effects. In the first step, a regression analysis was performed with aerobic exercise (*X*) as the independent variable and sleep quality (*Y*) as the dependent variable, and the regression coefficient *c* = −0.37 was obtained and reached the significance level to establish the regression equation *Y* = *F*[*X*, c, *τ*, *f*_*c*_, *ϕ*]. Using mental health as the dependent variable (*W*) and aerobic exercise as the independent variable (*X*), the regression coefficient was *a*_1_ = 0.14 and reached the significance level with an *F*-value of 6.79 (*P* < 0.001), and the standardized regression equation was *W* = *a*_1_*X* + *γ*. Mental health was the mediating variable between aerobic exercise and sleep quality, i.e., the mediating effect of mental health between aerobic exercise and sleep quality as a proportion of the total effect (−0.37x0.14/−0.46)∗100% = 11.26% [22]. The results suggest that the relationship between aerobic exercise and sleep quality is influenced by other factors besides mental health. Aerobic exercise negatively predicts sleep quality, aerobic exercise positively predicts mental health, and mental health negatively predicts sleep quality, which shows that each path of the model is significant, thus indicating that aerobic exercise can directly affect sleep quality and can also indirectly affect sleep quality through mental health. In other words, mental health plays a partially mediating role between aerobic exercise and sleep quality.

The article "Effects of Aerobic Exercise on Sleep Quality and Mental Health of College Students" was retracted in 2023. Reasons: signs of a paper mill; suspected computer-generated content; unreliable results or conclusions; lack of ethics approval or compliance.

### 3.4. Summary

According to the criteria for classifying exercise, a total score of >43 for exercise is considered heavy exercise, 20-42 for moderate exercise, and< 19 for small exercise. The results of this study show that the mean score for heavy exercise is 60.34 ± 14.86, accounting for only 8.5% of the total number of students, and the mean score for medium exercise is 28.66 ± 5.45, accounting for 16.0% of the total number of students, while the mean score of small exercise is 5.64 ± 6.53, accounting for 75.5% of the total number of students, indicating that the majority of college students have a small amount of daily aerobic exercise. The results of this study reflect the side that with the gradual increase of social pressure and the increasing development of modern information technology; the majority of college students need to spend more time on study, while their leisure time tends to be more devoted to the use of the Internet [23]. For example, male students like to play online games, and female students like to shop online and watch dramas, which leads to less time and time for exercise. The results of this study are similar to the results of existing studies; i.e., the percentage of small exercise (75.5%) is slightly higher than that of the previous study (70%), while the percentage of medium to large exercise (24.5%) is lower than that of the previous study (30%). Since there are relatively few studies of this type, it is not possible to make a more in-depth cross-sectional comparison.

Individuals with PSQI > 8 are considered to have sleep problems, and the higher the score, the worse the quality of sleep. The data from this survey showed that the total PSQI score of college students was 8.36 ± 2.59, which can be considered a poor quality of sleep for today's college students if the above-mentioned criteria for delineating the critical value of sleep quality are followed [24]. This study also found that the total PSQI score and the sleep time, sleep efficiency, subjective sleep quality, sleep disorder, and daytime dysfunction factor scores were higher than the reference values of sleep quality among college students. The reason may be that the social pressure faced by contemporary college students and the temptation brought by advanced electronic products take up more sleep time of individuals, which affects their sleep efficiency and daytime function, thus leading to the overall poor sleep quality for individuals [25]. However, there is a gap between the results of this study and similar studies in China.

The article "Effects of Aerobic Exercise on Sleep Quality and Mental Health of College Students" was retracted in 2023. Reasons: signs of a paper mill; suspected computer-generated content; unreliable results or conclusions; lack of ethics approval or compliance.

## 4. Discussion

In this study, we combined relevant theoretical explanations and evidence from previous empirical studies to test the mediating effect of mental health between aerobic exercise and sleep quality using the SPSS software, based on which we then used Amos to construct a model of the above three variables and summarize the relationship between the three variables. The structural equation model of this study presented the following characteristics [26]:

1. Aerobic exercise can directly affect sleep quality and influence various factors of sleep quality through mental health. The results showed that the lower the amount of aerobic exercise among college students, the worse their sleep quality
2. Aerobic exercise can directly affect mental health, indicating that the greater the amount of aerobic exercise of college students the higher their mental health
3. Mental health can directly affect the quality of sleep; i.e. the higher the mental health of college students, the better their sleep quality
4. Psychological health plays a partially mediating role in aerobic exercise and sleep quality; i.e., the individual's psychological health can weaken the effect of aerobic exercise on sleep quality, and maintaining a positive emotional state before bedtime can effectively promote the improvement of sleep quality among college students. According to the theoretical integration model in Figure 1, it can be seen that stimulation behavior can influence the level of individual emotional arousal, which in turn affects individual sleep quality

The results of this study show that mental health is a mediating variable between aerobic exercise and sleep quality. Existing college students have serious mental health and sleep quality problems, and there is an urgent need for schools to improve this problem by regulating the necessary aerobic exercise time for college students in the form of mandatory aerobic exercise classes.

## 5. Recommendation

To cultivate comprehensive and high-quality talents, the compulsory aerobics course is one of the important mandatory courses at the university level. Moreover, the relevant departments of colleges and universities should also make targeted programs according to the characteristics of students in the management of students. On the one hand, the compulsory aerobics courses in colleges and universities can set diversified types of sports according to the demographic characteristics of students, so that college students can make diversified choices according to their conditions [27]. Besides, relevant departments of colleges and universities should also actively promote extracurricular sports and carry out sports activities regularly or irregularly to encourage college students to integrate into the group and relieve the pressure of study and interpersonal aspects. On the other hand, relevant departments of universities should actively promote the issue of sleep hygiene and intervene in the formation of good sleep habits for students, for example, by controlling the time students' campus network use to urge them to form good sleep habits.

The article "Effects of Aerobic Exercise on Sleep Quality and Mental Health of College Students" was retracted in 2023. Reasons: signs of a paper mill; suspected computer-generated content; unreliable results or conclusions; lack of ethics approval or compliance.

## 6. Advantages and Limitations

In terms of research content, there are very few results combining aerobic exercise, mood, and sleep quality. The present study investigates the effects of aerobic exercise and emotion on sleep quality to fill this gap and provide empirical evidence for the theoretical basis. This study combines theories of kinesiology and psychology to analyze aerobic exercise, emotion, and sleep quality in depth and constructs a structural equation model between the three variables to explore the influence mechanism of sleep quality. In addition, we propose the necessity of mandatory aerobic exercise courses in universities and constructive suggestions based on the constructed model.

In terms of research methods, this study only used the sampling test method and questionnaire to study aerobic exercise, mood, and sleep quality among college students, which is too homogeneous. In addition, this study used a cross-sectional research method, so it was not possible to systematically determine the cross-sectional and longitudinal causal relationships among the variables.

## 7. Future Research Directions

Future studies can incorporate experimental research methods and use advanced research tools to explore the above three variables in depth. For example, a real-time tracking study of aerobic exercise was conducted on experimental subjects using relevant instruments, followed by observation of their brain imaging using various brain imaging techniques or monitors and a comprehensive assessment combined with relevant scales to improve the accuracy and scientific validity of the research findings. Future studies can add more possible factors to explore more deeply the mechanisms influencing the sleep quality of college students. In addition, there are relatively few studies on the relationship between aerobic exercise and sleep quality among college students, but the results of this study have demonstrated that aerobic exercise can predict sleep quality and that mood is a mediating variable between the two, and this conclusion is consistent with the existing theoretical explanations. Due to the limitations of the current research results, especially the small number of research instruments for aerobic exercise and the limitations of the research methods, the underlying mechanisms between the two need to be further explored in future studies. In this experiment, only experimental interventions were conducted for students in the experimental group, no experimental interventions were conducted for students in the control group, and only basic requirements were made without such strict monitoring as in the experimental group; it is suggested that the control group be included within the scope of monitoring during future experimental studies to make the intervention results of the experimental group more convincing.

The article "Effects of Aerobic Exercise on Sleep Quality and Mental Health of College Students" was retracted in 2023. Reasons: signs of a paper mill; suspected computer-generated content; unreliable results or conclusions; lack of ethics approval or compliance.

## 8. Conclusion

This study investigated the relationship between aerobic exercise and sleep quality and mental health of college students and further analyzed the pathway model of the effect of aerobic exercise and mental health on the sleep quality of students. The results of the study found that a 4-week period of moderate intensity was effective in improving the inhibition control of college students and that it improved both response inhibition and active inhibition. Some demographic variables, aerobic exercise, and sleep quality were also found to have significant effects on mental health and sleep quality, and mental health partially mediated the effect of aerobic exercise on sleep quality. The experiment was validated, and the need for a compulsory aerobic exercise course at university and other constructive suggestions was proposed.

## Figures and Tables

**Figure 1:** Graph of the association between aerobic exercise and physical and mental health.

**Figure 2:** Evaluation of response in the middle and late stages of exercise intervention.

**Table 1:** Sleep quality and descriptive analysis of each factor.

Variable	Human	Reference
Sleep quality	5.23 ± 0.6	5.41 ± 0.8
Time to fall asleep (min)	15 ± 10	12 ± 8
Sleeping time (h)	7 ± 2.5	8 ± 1
Hypnotic drugs	13.6% ± 3.8%	4% ± 1%
Sleep efficiency	73.1% ± 5.3%	80% ± 5%
Sleep disorder	6.9% ± 2.3%	5% ± 2%
PSQI score	16.25 ± 3.16	20 ± 5

**Table 2:** Distribution of subjects' basic conditions.

Variable	Variable characteristics	Number of people
Gender	Female	391
	Male	369

Health status	Healthy	283
	Good	261
	Bad	216

Aerobic exercise	Always	193
	Often	216
	Occasionally	164
	Hardly ever	137
	Never	40

The article "Effects of Aerobic Exercise on Sleep Quality and Mental Health of College Students" was retracted in 2023. Reasons: signs of a paper mill; suspected computer-generated content; unreliable results or conclusions; lack of ethics approval or compliance.

**Table 3:** Pre- and posttest comparisons of college students' mental health.

Test parameters	Variable characteristics	Number of people
Depression	Severe	56
	Mild	63
	None	641

Anxiety	Always	29
	Often	34
	Occasionally	53
	Hardly ever	314
	Never	330

Sensitive relationships	Yes	191
	No	569

Paranoia	Yes	237
	No	423

**Table 4:** Correlation analysis of aerobic exercise, mental health, and sleep quality among college students.

	Aerobic exercise volume	Sleep quality	Positive psychology	Negative psychology	PSQI score
Aerobic exercise volume	1	-0.34	0.67	-0.67	0.83
Sleep quality	-0.34	1	0.32	-0.34	0.61
Positive psychology	0.67	0.32	1	-1	0.71
Negative psychology	-0.67	-0.34	-1	1	-0.68
PSQI score	0.83	0.61	0.71	-0.68	1

## Data Availability

The data used to support the findings of this study are available from the corresponding author upon request.
